RETRACTED

# Exploration of the Visual Function after the Implantation of Continuous Visual Range Human Cocrystal Micromonocular Vision in Both Eyes of the Patient

**DOI:** 10.1155/2022/6000977

**Published:** 2022-03-07

**Authors:** Fangrong Cai, Xiaoli Wang, Zhihui Deng, Lina Bai

**Affiliations:** Ophthalmology, Jianyang People's Hospital, Jianyang 641400, China

## Abstract

Eye diseases such as myopia, hyperopia, astigmatism, and cataract are have affected most people at home and abroad for many years. With the development of science and technology, people who wear glasses are now younger, and they are on the rise over time. This paper is to explore the visual function after the implantation of continuous visual range human cocrystal micromonocular vision in both eyes of the patient. On this basis, the latest visual sensor technology is used to conduct clinical research on the operation, a case-control study is performed on the patient's eyes, followed by intraocular lens insertion surgery, one eye is hemitrope and the other eye has a certain degree of intraocular lens inserted, and it is recorded within a period of time after the operation. According to the analysis of the experimental results, the patient's naked eye and corrected distance vision is (t = 2.102, P = 0.049), middle distance vision (t = 1.403, P = 0.200), and near vision (t = 1.463, P = 0.216). After the operation, the ratio of patients taking off glasses 91.8%. After the continuous visual range intraocular lens micromonocular vision design, it can well correct the patient's near and far vision of the naked eye of both eyes.

## 1. Introduction

Nowadays, people's use of eyes is getting higher and higher, coupled with not paying attention to eye protection, leading to more and more occurrences of various eye diseases such as myopia, hyperopia, and astigmatism. Now myopia is becoming more and more popular. The eye population has been accounted for more than 50% of the national population, and there is a continuing upward trend over time. Monocular vision refers to a refractive state in which one eye sees the distance. A new type of contact lens can be designed for elderly patients to facilitate their use in life. To a certain extent, it provides patients with very satisfactory far and near vision. With the development of ophthalmic medicine, modern researchers have applied monocular vision in the treatment of ocular diseases, and it has been widely used in patients clinically. In the study, different methods were used to treat the two eyes differently. One eye was treated squarely according to the normal operation, and the other eye was implanted with a corresponding intraocular lens according to a certain diopter after the operation. Very satisfactory results have been achieved. Nanomaterials are materials that construct basic units of one- or three-dimensional space, and their scale is generally between 1 and 100 nm, roughly equivalent to the scale of 10 to 1,000 closely spaced atoms. After the intraocular lens implantation operation, the patient is tracked and observed, and the actual postoperative situation of the patient is recorded and fed back.

RETRACTED

The vision sensor is the direct source of information for the entire machine vision system. It is mainly composed of one or two graphic sensors, sometimes with light projectors and other types of auxiliary equipment. The main function of the vision sensor is to obtain enough original images to be processed by the machine vision system. After capturing the image, the vision sensor compares it with the reference image stored in the memory for analysis. For example, if the vision sensor is set to identify machine parts with eight bolts correctly inserted, the sensor knows that parts with only seven bolts should be rejected, or parts with misaligned bolts. In addition, no matter where the machine part is located in the field of view, whether the part is rotated within 360 degrees, the vision sensor can make a judgment. Using the vision sensor image in the operation, the specific conditions of the patient after the operation can be observed well, and the operation can be carried out more smoothly.

The far, intermediate, and near vision performance of patients implanted with a trifocal aspherical presbyopia correction intraocular lens (IOL) are evaluated. The defocus curve shows a wide range of useful vision. There are two best visual acuity peaks at a distance and 50 cm. The contrast sensitivity of the binocular distance is within the normal range. Alfonso J's vision performance obtained by bilaterally implanting the triple focal aspheric AcrySofIQ PanOptix IOL is good in far, medium, and near distances [1]. Central serous chorioretinopathy (CSCR) is a disease of unknown origin, which is characterized by macular serous detachment and affects young and healthy adults, mainly men aged 20–50. It is speculated that the Shrestha C study aims to evaluate the visual function test of CSCR after intravitreal bevacizumab injection [2]. In a randomized controlled trial, patients undergoing cataract surgery were bilaterally implanted with two different trifocal intraocular lenses (IOL) with similar optical zones but different tactile shapes. The visual results, rotational stability, and centrality of patients were evaluated and compared. The Poyales F study revealed similar visual results of the two tested trifocal intraocular lenses. However, the intraocular lens exhibits better rotational stability, as provided by its design [3]. Use objective image analysis techniques to determine the rotational stability of the Rayner 600S intraocular lens (IOL). Bhogal-Bhamra G K used the Rayner 600S intraocular lens to show excellent rotational stability and centrality after implantation, which meets the American National Standards Institute's standards for toric intraocular lenses specified by the US Food and Drug Administration [4]. An experiment was conducted to compare the visual effects and patient satisfaction of unilateral and bilateral trifocal diffractive intraocular lens (IOL) implantation in patients with emmetropia and presbyopia. The JL Fernández-García study has shown that RLE implanted with trifocal diffractive IOL in both eyes in patients with presbyopia is more successful than single-eye implantation in UNVA. However, no significant differences were observed in UDVA, UIVA, and patient satisfaction [5]. Based on the position experiment of the near and middle part of the eye with a rotationally asymmetric multifocal intraocular lens (IOL), the visual performance and high-order aberration (HOA) are compared. Song I S uses a rotationally asymmetric multifocal intraocular lens to have no significant effect on visual performance [6]. To evaluate the early detection of new single-focal intraocular lenses (Tecnis® Eyhance) and standard single-focal intraocular lenses (Tecnis® 1-piece) in patients undergoing cataract surgeries to standard single-focal intraocular lenses, Tecnis® Eyhance seems to be an effective choice for patients and surgeons because of its better intermediate vision and greater tolerance for residual refractive errors. Unsal U needs to conduct longer follow-up studies on more patients to evaluate the effectiveness of Tecnis® Eyhance intraocular lenses [7]. Compare the clinical results of a long-focus small-aperture intraocular lens (IOL) when implanted in one or both eyes to compensate for presbyopia. The bilateral implantation of the IC-8 intraocular lens expands the focus range and has a better near and medium vision. Implanting IC-8 IOL in a single eye can significantly improve the overall satisfaction score and lower aura score. Dick HB's bilateral implantation of IC-8 IOL leads to an enlarged focal range, which has better mid- and near-sight vision than monocular implantation of the IOL [8]. However, the above research did not propose a new type of intraocular lens material. The traditional intraocular lens has many shortcomings, which will make it difficult to recover after surgery. It will also need to be replaced within a period of time, and many clinical trials have not been carried out. On further inquiry, there is a lack of specific theoretical support at the theoretical level.

RETRACTED

Silicon gel is one of the commonly used materials for intraocular lenses. The soft intraocular lens produced has been used at home and abroad before, and it is also one of the lenses that have been used clinically. It has the characteristics of low specific gravity, high temperature resistance, high pressure resistance, and so on. It is not easy to age under high temperature, so it can be sterilized by high pressure or boiling, but the silicone gel material is easy to adhere to particles, which will affect its transparency and light transmittance, and long-term use may damage the lens. The intraocular lens designed using new nanomaterials has the characteristics of not easy to absorb smell, sterilization, and high temperature resistance. Compared with traditional materials, it is not easy to absorb particulate matter, will not absorb eye secretions, and will not affect the intraocular lens implanted in the eyeball. When damaged, it is possible to carry out the continuous vision intraocular lens micromonocular design operation, that is, the intraocular lens implantation operation, and it will not have other effects on the patient in the later recovery and normal life.

## 2. Observation Method of Visual Function after Intraocular Lens Micromonocular Design

### 2.1. Vision Sensor

The vision sensor is the direct source of information for the entire machine vision system. It is mainly composed of one or two graphic sensors, sometimes with light projectors and other types of auxiliary equipment. The main function of the vision sensor is to obtain enough original images to be processed by the machine vision system. The image sensor can be a laser scanner, a linear and area CCD camera or a TV camera, or the latest digital camera. The sensor system is shown in Figure 1.

Machine vision is widely used in medical production and is commonly used in four types of functions: visual guidance and positioning, pattern recognition and detection, precise measurement and distance measurement, and medical detection. In a nutshell, the feature of medical machine vision system is to improve the flexibility and automation of production, mainly in some dangerous working environments that are not suitable for manual work or occasions where artificial vision is difficult to meet the requirements, and machine vision is used to replace artificial vision. The medical vision application and its requirements for sensor parameters are shown in Figure 2.

Nanomaterials refer to materials manufactured in the traditional three-dimensional space with a size of 1–100 nm as the basic unit, which is equivalent to the length of 10–1000 atoms arranged together at the atomic level [9]. With the gradual development of nanomaterials, many cooperation projects and applications related to nanomaterials have made great breakthroughs. Nanomaterials have begun to be used in all walks of life because of their high melting point, good magnetic properties, and electrical and thermal conductivity. When the size of nanomaterials is within a certain range, they cannot be manufactured by traditional technology [10]. When the particle size of the powder is reduced from 10 microns to 10 nanometers, even if the particle size of the nanomaterial is converted to 1000, the volume is 10 to the ninth power, so the behavior of the two is obviously different. Nanostructured materials are referred to as nanomaterials. This means that the size of the building unit ranges from 1 nm to 100 nm because its size is close to the length of the relevant electron. Therefore, due to the self-organization caused by strong cohesion, its properties have changed a lot. After all, its scale is close to the wavelength of light, combined with the special effects of large textures and the performance characteristics of the substance in its overall state [11]. With the development of the times, nanomaterials are widely used in medical, nanocomputer, environment, and so on and have achieved good results.  Figure 3 shows the application scope of nanomaterials.

RETRACTED

In the field of nanotribology, that is, in the field of nanobiology, in nanoscale phenomena, atomic interaction and quantum influence cannot be ignored [12]. For example, the purpose of appearance research is to clarify and verify the surface properties of materials from the basic properties and applications of materials. In traditional nanotribological research, only direct research has been carried out, with very high-resolution experiments, and surface characteristics, such as scanning tunneling microscope (STM), atomic force microscope (AFM), surface force device (SFA), and various microscopic methods, have been observed. Due to the development of calculation methods and the efficiency of computers, what can be analyzed now plays an important role [13]. Therefore, computational science methods can be used for research. From the macroscopic study of sliding friction, the friction formula can be obtained; that is, the friction force F is proportional to the load *P*, and the friction coefficient proportional constant is *μ*.

(1) $$\begin{array}{c} F=\mu P. \end{array}$$

The friction force of the adhesive contact surface is the friction force of the interface, and the friction force is the necessary resistance to overcome the shear force at the adhesive joint [14].

(2) $$\begin{array}{c} F=\tau_{c}A, \end{array}$$

where *A* is the contact area with the adhesive, calculated according to the specified elastic contact type JKR, and taking into account the effect of the adhesive energy on the surface, for the hemisphere with radius *r* tangent to the plane, the relationship between the contact area A and the load *P* is

(3) $$\begin{array}{c} \frac{A}{A_{0}}={\left\{\frac{1}{2}\left[\left(1+\frac{y}{2}\right)+{\left(1+y\right)}^{1/2}\right]\right\}}^{2/3}, \end{array}$$

(4) $$\begin{array}{c} y=\frac{-P}{P_{s}}, \end{array}$$

(5) $$\begin{array}{c} P_{s}=3\pi r\omega . \end{array}$$

The surface force instrument SFA was used to carry out relevant experimental studies on the friction characteristics of the interface of mica materials. Two different mica sheets adhered to the surface of a cylinder made of two silica gel materials, and the two cylinders were orthogonal zed. Placement can increase the friction of the contact point, and the contact area is a regular circle, simulating the contact situation of a single rough peak [15]. The experimental results show that when the surface is sliding under the condition of molecular contact, the ultimate shear force should be composed of three parts.

(6) $$\begin{array}{c} \tau_{\text{c}}=\tau_{c_{1}}+\tau_{c_{2}}+\tau_{c_{3}}. \end{array}$$

By quoting the relevant relational expression in Hentz's elastic contact theory, we can see that equation (6) can be rewritten as

(7) $$\begin{array}{c} F=C_{1}P^{2/3}+C_{2}P+C_{3}P^{4/3}. \end{array}$$

The preparation of nanomaterials currently prevailing at home and abroad generally includes the sol-gel method, in situ polymerization method, blending method, and template method. Among them, the template synthesis method uses nanostructured materials and easy-to-use shapes, and this material is cheap and easy to find as a template. Put the corresponding physical or chemical material into the hole or surface of the template, and then take out the template to obtain the template with the standard morphology of the nanomaterial size [16]. The simulation method is also one of the important methods for the synthesis of nanocomposite materials. It is also the most widely used method for studying nanomaterials, especially in the production of nanomaterials with unique properties. The template method can design standard materials according to the performance and morphological requirements of synthetic materials and structures to meet actual needs. The template synthesis method is an effective method for preparing nanomaterials. The main feature is that the template synthesis method is a chemical reaction that occurs in the liquid phase or the gas phase. The reaction occurs in an effectively controlled area. This is a standard method, which is compared with the traditional method.  Figure 4 shows the nanostructured material prepared by the template synthesis method.

RETRACTED

### 2.2. Micromonocular Design of Intraocular Lens

Intraocular lens micromonocular vision design surgery is intraocular lens surgery. Putting the intraocular lens into the eyeball through surgery can improve the visual condition to a certain extent [17]. Intraocular lens is currently the most effective way to correct blurred vision. It replaces the original anatomical and optical lenses. By creating an almost normal system, especially the artificial rear groove lens installed in the normal position of the normal lens, each eye can be used, the vision can be quickly restored after the operation, and it is easy to establish binocular monovision and stereo vision [18]. Since Ridley, a well-known British ophthalmologist, discovered a suitable intraocular lens material in 1949, after many generations of development, many intraocular lens materials have been discovered, which can produce intraocular lenses that are very in line with the physiological state of humans and can be used for human eyeballs. And there are very mature treatments for surgery now [19]. The intraocular lens micromonocular design is to remove the cloudy lens and then implant the intraocular lens to achieve the effect of restoring vision. It has the advantages of fewer complications, faster healing, and faster vision recovery. It can bring different postoperative visual effects to patients and achieve a more perfect visual quality.  Figure 5 shows the specific implantation operation for this operation.

The initial preparations for intraocular lens surgery require the calculation of the degree of the intraocular lens. The development process of this formula is from the initial experience to the original theoretical formula. After a period of research and development, the formula is developed. The first-generation formula is the ideal model, and the second and third-generation formulas that were subsequently developed have gradually adapted to the inquiry into the degree of intraocular lens required in this era [20]. The empirical theoretical level is

(8) $$\begin{array}{c} IOL=18+\left(R\times 1.25\right). \end{array}$$

The original theoretical formula proposed by the predecessor scientists based on the accumulation of long-term experience is an epoch-making theory and has laid a solid foundation for subsequent research on related formulas:

(9) $$\begin{array}{c} P=\frac{n}{\left(L-c\right)}-\frac{n}{\left[\left(n/K\right)-c\right]}, \end{array}$$

where *P* is the power of the intraocular lens, *L* is the axial length of the eye, *c* is the estimated depth of the anterior chamber, *K* is the curvature of the cornea, and *n* is the relative refractive index of the eye chamber and the vitreous.

RETRACTED

The SRK/T formula is a third-generation formula based on the Fyodorov formula, where the prediction formula of *c* is

(10) $$\begin{array}{c} c=H+offset, \end{array}$$

(11) $$\begin{array}{c} offset=0.62A-\partial \cdot \theta -3.36, \end{array}$$

where *H* is the actual distance from the cornea to the iris plane and ∂·*θ* is the ideal distance from the cornea to the iris plane.

In the Holladay and Holladay 2 formulas, the prediction formula of *c* is

(12) $$\begin{array}{c} ELP=aACD+S, \end{array}$$

(13) $$\begin{array}{c} aACD=0.56+R{\left[R^{2}-{\left(AG\right)}^{2}\left(\frac{1}{4}\right)\right]}^{-2}, \end{array}$$

(14) $$\begin{array}{c} AG=L\times 12.5\times \left(\frac{1}{23.45}\right), \end{array}$$

(15) $$\begin{array}{c} S=A-cons\;\tan\;t\times 0.56-65\partial . \end{array}$$

Among them, *aACD* represents the depth of the anterior chamber of the eye before the operation, *S* represents the distance from the anterior surface of the iris to the optical plane of the intraocular lens, *R* is the radius of curvature of the cornea, and *AG* is the diameter of the anterior chamber of the eye.

There are two classifications of intraocular lenses. One is based on the specific fixed position of the intraocular lens in the eye. There are anterior chamber intraocular lenses and posterior chamber intraocular lenses in this category. There will be many complications after the operation, which may be dangerous to the patient, so most of the operations currently performed are posterior chamber intraocular lens implantation [21]. The other is divided according to different materials. Polymethyl methacrylate is the first material used to make intraocular lenses and the material of choice for hardening intraocular lenses. It has stable performance, light weight, and good transparency and will not be degraded by the body's biological oxidation reaction. But the disadvantage is that it cannot withstand high temperature and high pressure sterilization. At present, ethylene oxide is used for disinfection, and its flexibility is low. There are two types of clinical applications: one is an intraocular lens made of PMMA material at the same time, called the one-piece type; the other is that the optical part and ring of the lens made of PMMA material are made of polypropylene; silicone gel is now the main material for the soft intraocular lens, with high temperature resistance, good thermal stability, antiaging, good biocompatibility, and so on, but the shortcomings are also very obvious, poor toughness, easy to generate static electricity, and very easy to absorb some dust and other things. Hydrogel is a very popular hydrophilic material. It has the characteristics of good stability, good compatibility, and high strength. However, because of its rich water permeability, it is easy to attach substances to the eyes, which will affect the transparency; acrylic acid the ester is composed of phenylethyl acrylate and phenylethyl methacrylate, which is a copolymer with optical and biological properties equivalent to PMMA. It has the characteristics of strong flexibility, small size, and elasticity [22].  Figure 6 shows the specific classification of intraocular lenses.

RETRACTED

### 2.3. Postoperative Observation of Intraocular Lens Micromonocular Design

Intraocular lens refers to a special lens made of artificial synthetic materials. The composition includes silica gel, polymethyl methacrylate, and hydrogel. The shape and function of the lens of the eye are similar to those of the human eye. It is light in weight and has good visual properties. It is nonantigenic, inflammatory, carcinogenic, and biodegradable [23]. Remove the blurred lens after eye surgery. An intraocular lens is implanted in the eye to replace the original lens. This makes it possible to focus and photograph foreign objects in the retina and to clearly see the surrounding landscape to reduce the recurrence of eye diseases after intraocular lens surgery. Generally, surface modification of intraocular lens materials is used to reduce the adhesion of lens epithelial cells. The proliferation and remodeling of lens epithelial tissue can also be achieved by blocking drugs [24]. As shown in Figure 7, it is now possible to process and modify the surface of the intraocular lens material to obtain a hydrophilic surface mucosa, thereby inhibiting the adhesion of lens epithelial cells, which can greatly increase the occurrence of eye diseases.

Since the first posterior chamber intraocular lens (PCP ICL) implantation operation was performed to correct human vision problems in 1986, the technology has been widely used worldwide and is used by relevant personnel from all over the world. Carry out in-depth research and vigorously develop related technical techniques [25]. The biggest advantage of using this intraocular lens surgery is that it does not make any changes to the patient's ocular structure. There are some areas that cannot be reached in traditional surgical operations. The use of intraocular lens surgery can operate on areas that cannot be covered by traditional surgery [26–28]. It has become the preferred treatment method for the treatment of human vision problems in clinical practice and has been widely used by relevant institutions at home and abroad.  Figure 8 shows the process of observing the patient after the intraocular lens implantation operation, including some preoperative and postoperative follow-up care of the patient, including a detailed understanding of the patient's details before the operation. Record the patient's physical and psychological status; during the operation, the nurse should help the doctor, observe the patient's situation in real time, and give feedback in time; after the operation, it is necessary to observe the patient's postoperative situation, timely give feedback to the chief physician, and actively respond to the actual situation of the patient shall be dealt with accordingly, and targeted training shall be carried out in the later rehabilitation of the patient.  Figure 8 presents preoperative and postoperative care during intraocular lens surgery.

RETRACTED

## 3. Observation Experiment of Visual Function after Continuous Visual Range Intraocular Lens Micromonocular Design

### 3.1. Design Surgery of Intraocular Lens Micromonocular Vision

Intraocular lens micromonocular vision design surgery involves implanting the intraocular lens into the posterior chamber of the eye, the iris, and the area between the lenses behind the eyeball. It can correct several eye symptoms, such as myopia, hyperopia, and astigmatism, without removing or splitting. Destroy the cornea and other tissues, and do not need to suture after the operation. It is one of the very fast, convenient, and effective eye surgeries. The monocular vision design places the patient's one eye to look squarely after the operation while the other eye is implanted with an intraocular lens. All operations are performed by the same expert who has been doing this operation for many years. A 2 mm transparent corneal incision should be made for the surgical eye to facilitate the implantation of the intraocular lens. After the operation, the cloudy lens should be sucked out, the viscoelastic agent should be sucked out, and the incision should be water tightly closed. The results after the operation are shown in Table 1. The distance vision of the emmetropia designed by the patient meets the standard requirements, the near vision of the design myopia also meets the requirements, and the myopia is far better than the emmetropia. Both naked eyes can produce satisfactory results at long distances, middle distances, and short distances. Table 1 is a comparison of naked eyes and corrected visual acuity for a period of time after the operation.

RETRACTED

After the operation, the patients in the photopic and scotopic environment are compared. Within the frequency space range of the photopic condition, the sensitivity of the eyes in the uncorrected state is lower than the sensitivity of the eyes after correction; in the scotopic condition, the contrast between the sensitivity of the uncorrected binocular and the sensitivity of the corrected binocular in each frequency space range below is roughly the same as that under the photopic conditions, but the difference between them is not statistically significant.  Table 2 shows the comparison of the sensitivity of both eyes with naked eyes and after correction in the range of the photopic space within a period of time after surgery.

Table 3 shows the comparison of the sensitivity of both eyes with naked eyes and after correction in the scotopic space for a period of time after the operation.

### 3.2. Observation of the Situation before Surgery

A detailed understanding is done of the age, visual acuity, intraocular pressure, and the degree of intraocular lens implantation of the three groups of patients, statistics of the specific data of each patient for comparison, and the use of SPSS 23.0 statistical software for data collection. If the measurement data obey the normal distribution, the collected three groups of patients data *χ*^2^ are used to test the gender. If the measurement data do not meet the normal distribution, the paper compares multiple groups and uses multiple independent samples to sort the test. The statistical differences are shown in Table 4.

Perform detailed follow-up observations within a period of time after the implantation of the intraocular lens, check the recovery of the patient after the operation, compare the patient's uncorrected distance vision with the best corrected distance vision, and compare them at 3 months and 6 months after the operation. A detailed comparison of the two visual acuities of the month showed that the differences between the three groups of patients were not detailed and not statistically significant. The specific conditions are shown in Table 5.

During a period of time after the lens implantation operation, the patients were tracked to observe the recovery, and the intermediate visual acuity of the three groups of patients was compared. The difference between them is based on the actual statistical significance. After multiple comparisons between the different groups, it is found that the intermediate visual acuity of the Z group and R group is lower than that of the T group, and the difference between them is statistically significant. However, the comparison between the Z group and the R group shows that their difference is not statistically significant.  Figure 9 shows the comparison of intermediate vision within a period of time after intraocular lens implantation surgery.

RETRACTED

Figure 10 shows the comparison of UCNVA and DCNVA of the three groups of patients. The difference between them is statistically significant. However, a multiple comparison between the different groups found that the R group and the Z group are higher than the T group. Comparing the R group with the Z group, the difference between them is statistically significant.

### 3.3. Sensitivity after Intraocular Lens Surgery

After the intraocular lens surgery, the patients were followed up for a period of time. In the bright environment, the frequency CS of the three groups of patients was compared within 3 and 6 months after the surgery. The difference between them was not statistically significant. Significance: under dark conditions, the three groups of patients were compared with each spatial frequency within 3 and 6 months after surgery. The comparison between CSs at 3c/d was not statistically significant. While at 6c/d, 12c, the comparison between CS at /d and 18c/d is statistically significant. As shown in Figure 11, multiple comparisons between different groups found that the R group has the lowest value and the T group has the highest value, and the difference between them is statistically significant.

In the glare environment, follow up for a period of time after the intraocular lens implantation operation. In the 3 months and 6 months after the operation, the CSs of the three groups at the spatial frequency of 3c/d were compared. There is no specific statistical significance, and the comparison of CS with spatial frequencies of 6c/d, 12c/d, and 18c/d has specific statistical significance. After multiple comparisons between different groups, it is found that the R group has the lowest value, the Z group is in the middle, and the value of the T group is the highest. The difference between them has specific statistical significance, as shown in Figure 12.

## 4. Discussion

In the traditional treatment of myopia, hyperopia, astigmatism, and other eye diseases, the two eyes of the patient are usually not operated on at the same time. After the lens, the balance of the eyes will be corrected in terms of the refractive power of the lens. However, after the single-focal intraocular lens is implanted in the eyeball, the patient's distance vision needs to be added nearby. As people use their eyes more and more frequently and now people are paying more and more attention to the protection of their eyes. The eyes are the windows of the soul. The comprehensive restoration and reconstruction of functional vision reduce the dependence on glasses. Now the main clinical application is the single focus lens, so the related methods of monocular vision design can be widely used in clinical practice. This experiment is to use vision sensor image technology for continuous visual range intraocular lens micromonocular vision design to conduct in-depth research on visual function after design. The contrast sensitivity of the two eyes in the uncorrected state under the spatial frequency of photonic and scotopic vision is studied. It is found that the sensitivity in the uncorrected state is slightly lower than that after the correction, which may be caused by the problem of the experimental operation, and the difference between the two is not statistically significant. It can be basically judged through experiments that the monocular lens design can generally meet the clinical needs of patients to remove the glasses, but due to anisometropia, stereo vision is significantly impaired after surgery, and subjective adjustment procedures are required. Although daily activities related to depth perception and stereo vision cannot be used for long-term monitoring, it is quite difficult to receive patients before surgery. According to research, the main factor affecting the success of vision is not postoperative stereo vision or other objective indicators of visual function, but the preoperative monocular vision of the patient is subjectively accepted. Therefore, the design of monocular vision surgery has certain clinical significance.

RETRACTED

## 5. Conclusions

Traditional intraocular lenses use silicone gel as a material for the development of soft intraocular lenses and are widely used in clinical trials. However, it is very easy to adhere to particulate objects such as dust and can easily damage the eyeball after surgery. The use of a new type of vision sensor image technology can be well designed to track related surgical procedures in the experiment and can be well applied in the tracking and observation of patients after surgery. In the uncorrected state, the sensitivity of the naked eyes of both eyes at spatial frequencies such as photonic and scotopic vision is lower than that of the naked eyes in the corrected state. From the results of the study, it can be judged that the monocular design of the continuous visual range intraocular lens micromonocular design can well meet the clinical needs of patients with ocular diseases. However, due to the operation of the original lens, it will have a certain impact on the patient's stereo vision after surgery. It needs to be observed, recovered, and adopted within a period of time after the surgery. It also needs to be reexamined in the hospital for a long time to eliminate the impact on the patient's normal life. As for patients with vision problems, this monocular design has very important clinical significance.

RETRACTED

## Figures and Tables

**Figure 1:** Sensor system diagram.

**Figure 2:** Medical vision application and its requirements for sensor parameters.

**Figure 3:** Specific application industry scope of nanomaterials.

**Figure 4:** Preparation of nanostructured materials by template synthesis.

**Figure 5:** Specific operation of intraocular lens surgery. (a) Shatter the turbid lens. (b) Aspirate the crushed lens. (c) Implant the intraocular lens.

**Figure 6:** Specific classification of intraocular lenses.

**Figure 7:** Technology based on genotype intraocular lens and its preparation method.

**Figure 8:** Preoperative and postoperative care during intraocular lens surgery.

**Figure 9:** Comparison of intermediate visual acuity within a period of time after the operation of the three groups of patients.

**Figure 10:** Comparison of UCNVA and DCNVA within a period of time after the operation of the three groups of patients.

**Figure 11:** Comparison of contrast sensitivity of three groups of patients in bright environment.

**Figure 12:** Contrast sensitivity in glare environment for a period of time after the operation of the three groups of patients.

**Table 1:** Comparison of naked eyes and corrected visual acuity for a period of time after the operation.

	Distance vision	Medium vision	Near vision
Naked eye	0.69 ± 0.14	0.54 ± 0.06	0.54 ± 0.20
Correct	0.80 ± 0.15	0.44 ± 0.05	0.57 ± 0.09
*t* value	2.102	1.403	1.463
*P* value	0.049	0.200	0.216

**Table 2:** Comparison of the sensitivity of both eyes with naked eyes and after correction within the range of the photopic space for a period of time after surgery.

	1.5	3.0	6.0	12.0	18.0
Naked eye	1.54 ± 0.34	1.49 ± 0.41	1.14 ± 0.78	0.66 ± 0.39	0.10 ± 0.09
Correct	1.54 ± 0.49	1.58 ± 0.59	1.20 ± 0.59	1.03 ± 0.59	0.12 ± 0.30
*t* value	1.27	0.69	0.31	1.60	1.12
*P* value	0.31	0.51	0.80	0.14	0.41

**Table 3:** Comparison of the sensitivity of both eyes with naked eyes and after correction within the range of the photonic space for a period of time after surgery.

	1.5	3.0	6.0	12.0
Naked eye	1.31 ± 0.49	1.10 ± 0.53	1.18 ± 0.59	0.34 ± 0.41
Correct	1.40 ± 0.61	1.55 ± 0.59	1.21 ± 0.68	0.59 ± 0.39
*t* value	0.759	1.734	1.103	1.692
*P* value	0.657	0.147	0.162	0.079

**Table 4:** Comparison of the general conditions of the three groups of patients before surgery.

	Age	Preoperative vision	Intraocular pressure	Implantation of intraocular lens power
Group T	65.17 ± 4.35	0.14 ± 0.08	14.98 ± 1.15	21.04 ± 1.12
Group R	64.57 ± 3.45	0.15 ± 0.06	14.94 ± 1.32	18.92 ± 0.79
Group Z	63.58 ± 3.27	0.17 ± 0.05	15.04 ± 1.57	20.04 ± 0.75
Group P	0.059	0.204	0.203	0.090

RETRACTED

**Table 5:** Comparison of uncorrected visual acuity and corrected distance visual acuity within a period of time after the operation of the three groups of patients.

	3 months after surgery		6 months after surgery	
	UCDVA	BCDVA	UCDVA	BCDVA
Group T	0.67 ± 0.15	0.89 ± 0.09	0.69 ± 0.12	1.01 ± 0.08
Group R	0.80 ± 0.16	0.90 ± 0.12	0.82 ± 0.15	0.90 ± 0.10
Group Z	0.71 ± 0.14	0.98 ± 0.10	0.75 ± 0.14	0.95 ± 0.07
Group P	0.498	0.408	0.248	0.624

## Data Availability

The simulation experiment data used to support the findings of this study are available from the corresponding author upon request.

## References

[1] Alfonso J. F., Fernández-Vega-Cueto L., Fernández-Vega L., Montés-Micó R. (2020). Visual function after implantation of a presbyopia-correcting trifocal intraocular lens. *Ophthalmic Research*.

[2] Shrestha C., Shrestha S., Manoranjan A. (2019). Evaluation of Visual Function Test of Central Serous Chorioretinopathy After Intravitreal Bevacizumab. *Medical Journal of Shree Birendra Hospital*.

[3] Poyales F., Garzón N., Rozema J. J., Romero C., de Zárate B. O. (2016). Stability of a novel intraocular lens design: comparison of two trifocal lenses. *Journal of Refractive Surgery*.

[4] Bhogal-Bhamra G. K., Sheppard A. L., Kolli S., Wolffsohn J. S. (2019). Rotational stability and centration of a new toric lens design platform using objective image analysis over 6 months. *Journal of Refractive Surgery*.

[5] Fernández-García J. L., Llovet-Rausell A., Ortega-Usobiaga J. (2021). Unilateral Versus Bilateral Refractive Lens Exchange With a Trifocal Intraocular Lens in Emmetropic Presbyopic Patients. *American Journal of Ophthalmology*.

[6] Song I. S., Yoon S. Y., Kim J. Y., Kim M. J., Tchah H. (2016). Influence of near-segment positioning in a rotationally asymmetric multifocal intraocular lens. *Journal of Refractive Surgery*.

[7] Unsal U., Sabur H. (2021). Comparison of new monofocal innovative and standard monofocal intraocular lens after phacoemulsification. *International Ophthalmology*.

[8] Dick H. B., Elling M., Schultz T. (2018). Binocular and monocular implantation of small-aperture intraocular lenses in cataract surgery. *Journal of Refractive Surgery*.

[9] Rosen E., Alió J. L., Dick B. H., Dell S., Slade S. (2016). Efficacy and safety of multifocal intraocular lenses following cataract and refractive lens exchange: Metaanalysis of peer-reviewed publications. *Journal of Cataract and Refractive Surgery*.

[10] Eom Y., Song J. S., Kim H. M. (2017). Spectacle plane add power of multifocal intraocular lenses according to effective lens position. *Canadian Journal of Ophthalmology*.

RETRACTED

[11] Alfonso J. F., Fernández-Vega Cueto L., Belda-Salmerón L., Montés-Micó R., Fernández-Vega L. (2016). Visual function after implantation of a diffractive aspheric trifocal intraocular lens. *European Journal of Ophthalmology*.

[12] Liu M. M., Dai J. M., Liu W. Y., Zhao C. J., Lin B., Yin Z. Q. (2016). Human melanopsin-AAV2/8 transfection to retina transiently restores visual function in rd1 mice. *International Journal of Ophthalmology*.

[13] Pineles S. L., Chen M. F., Velez F. G., Mathern G. W. (2018). Visual function after cerebral hemispherectomy. *Journal of American Association for Pediatric Ophthalmology and Strabismus*.

[14] Heo W., Kim J. S., Chung C. K., Lee S. K. (2017). Relationship between cortical resection and visual function after occipital lobe epilepsy surgery. *Journal of Neurosurgery*.

[15] Nguyen J. H., Nguyen-Cuu J., Yu F. (2019). Assessment of Vitreous Structure and Visual Function after n Laser Vitreolysis. *Ophthalmology*.

[16] Ferreira-Ríos I., Zuñiga-Posselt K., Serna-Ojeda J. C., Chávez-Mondragón E. (2018). Objective and subjective results following implantation of the FineVision trifocal intraocular lens in Mexican patients. *International Ophthalmology*.

[17] Rementería-Capelo L. A., Contreras I., García-Pérez J. L., Blázquez V., Ruiz-Alcocer J. (2019). Visual quality and patient satisfaction with a trifocal intraocular lens and its new toric version. *Journal of Cataract & Refractive Surgery*.

[18] Benck J. D., Hellstern T. R., Kibsgaard J., Chakthranont P., Jaramillo T. F. (2014). Catalyzing the hydrogen evolution reaction (HER) with molybdenum sulfide nanomaterials. *ACS Catalysis*.

[19] Rzayev J. (2017). Molecular Bottlebrushes: New Opportunities in Nanomaterials Fabrication. *ACS Macro Letters*.

[20] Luo Q. H., Liu B., Chen L. (2021). The effects of posterior chamber intraocular lens implantation on accommodative function in high myopia. *Chinese Journal of Ophthalmology*.

[21] Kohnen T., Lwowski C., Hinzelmann L. (2020). Presbyopia correction in astigmatic eyes using a toric trifocal intraocular lens with quadrifocal technology. *Journal of Refractive Surgery*.

[22] Bhalla M., El-Haddad O., Maurino V. (2020). Opacified hydrophilic intraocular lens following DMEK. *Eye*.

[23] Mano F., LoBue S. A., Eno A., Chang K.-C., Mano T. (2020). Impact of posterior vitreous detachment on contrast sensitivity in patients with multifocal intraocular lens. *Graefe’s Archive for Clinical and Experimental Ophthalmology*.

[24] Khler J., Khler K., Khler J. (2020). Primre hintere Kapsulorhexis in schwierigen Situationen. *Ophthalmologe, Der*.

RETRACTED

[25] Rong X., Miao A., Yu J. (2019). Case series: slight Intraocular lens malpositioning as a potential cause of vision loss. *Optometry and Vision Science*.

[26] Zhang Q., Zhou C., Tian Y. C., Xiong N., Qin Y., Hu B. (2017). A fuzzy probability Bayesian network approach for dynamic cybersecurity risk assessment in industrial control systems. *IEEE Transactions on Industrial Informatics*.

[27] He R., Xiong N., Yang L. T., Park J. H. (2011). Using multi-modal semantic association rules to fuse keywords and visual features automatically for web image retrieval. *Information Fusion*.

[28] Wei W., Zhou B., Połap D., Woźniak M. (2019). A regional adaptive variational PDE model for computed tomography image reconstruction. *Pattern Recognition*.

